# Computational Intelligence Based Recurrent Neural Network for Identification Deceptive Review in the E-Commerce Domain

**DOI:** 10.1155/2022/4656846

**Published:** 2022-11-18

**Authors:** Saleh Nagi Alsubari, Theyazn H. H. Aldhyani, Sachin N. Deshmukh, Mashael Maashi, Sadeen Alharbi, Heyam H. Al-Baity

**Affiliations:** ^1^Department of Computer Science & Information Technology, Dr. Babasaheb Ambedkar Marathwada University, Aurangabad, India; ^2^Applied College in Abqaiq, King Faisal University, P.O. Box 400, Al-Ahsa 31982, Saudi Arabia; ^3^Software Engineering Department, College of Computer and Information Sciences, King Saud University, Riyadh 11543, Saudi Arabia; ^4^Information Technology Department, College of Computer and Information Sciences, King Saud University, Riyadh, Saudi Arabia

## Abstract

Most consumers depend on online reviews posted on e-commerce websites when determining whether or not to buy a service or a product. Moreover, due to the presence of fraudulent (deceptive) reviews, the fundamental problem in such reviews is not fully addressed. Thus, deceptive reviews present wrong and misguiding opinions that are harmful to consumers and e-commerce. People called fraudsters who intentionally write deceptive reviews to target and deceive potential consumers, as they target businesses that have a well-built reputation or fame for their personal promotion, create such reviews. Therefore, developing a deceptive review detection system is essential for identifying and classifying online product reviews as truthful or fake/deceptive reviews. The main objective of this research work is to analyze and identify online deceptive reviews in electronic product reviews in the Amazon and Yelp domains. For this purpose, two experiments were conducted individually. The first was executed on standard Yelp product reviews. The second was performed on Amazon product review datasets. For this dataset, we created and labeled it using a deceptiveness score calculated based on features extracted from the review text using the linguistic inquiry and word count (LIWC) tool. These features were authenticity, negative words, comparing words negation words, analytical thinking, and positive words as well as the given rating value by a user. The recurrent neural network, bidirectional long short-term memory (RNN-BLSTM) model, was used to both datasets in order to conduct the evaluation. The application of this model was contingent upon the learning of words embedding of the review text. Finally, we evaluated the RNN-BLSTM model's performance using the Yelp and Amazon datasets and compared the results. The results were 89.6% regarding testing accuracy for both datasets. From our experimental results, we observed that the LIWC feature with word embedding in the review text provided better accuracy performance compared with other existing methods.

## 1. Introduction

The advance of Web 4.0 has improved the activity of online marketing by using e-commerce sites. Customer reviews produced in e-business websites and social networks indicate the perception of consumers. Therefore, such reviews play an important part in e-business as they may remarkably affect buying decisions due to the existence of deceptive reviews that offer false and misleading opinions that do not represent the honest product experience of a customer. These reviews can be posted and released on many online shopping sites, such as Amazon, Yelp, TripAdvisor, Flipkart platforms, and other websites [1]. In general, the number of users of these sites has increased over the last few years. Nowadays, when consumers acquire online products or services, they search for reviews posted by customers who have previous experience with the products [2]. Manufacturers of products utilize consumer's competitors to discover the defects in the e-commerce products and to collect market-intelligent information regarding their opponents. Using online reviews to leverage the judging capacity of product/service quality, fraudsters produce fake feedback called fake reviews. Not all reviews posted on e-commerce websites are truthful reviews; the ratio of fake reviews varies from 16% to 33.3% [3, 4]. Around 10.3% of online items have been exposed to review manipulation [5]. Fake reviews are classified into the following three types: First, untruthful reviews that are intentionally generated to trick users or opinion-mining systems are known as incorrect (false) reviews. These reviews include irrelevant affirmative feedback regarding the product or service to particular target markets. In addition, they provide misleading feedback to defame deserving products. Second, reviews on a company name only are reviews that focus on the brand of producers or sellers, but not on the product itself. Finally, nonreviews are reviews that do not contain opinions, such as inquiries, responses, or unspecified topics. Non-feedbacks or evaluations have two subsets: (a) commercials and advertisements; (b) unconnected reviews [6]. Most marketplaces prefer well-evaluated goods, potentially rewarding companies that pay for false reviews. Vast amounts of positive reviews motivate buyers to purchase and boost manufacturers' business profits, while destructive (negative) reviews allow consumers to explore and look for alternatives, leading to financial losses [7]. Identifying and differentiating fake reviews from trusted ones can also be difficult because of the number of reviews released online and the skills of review fraudsters. Moreover, detecting and removing such reviews from review websites and product recommender systems are important for businesses and consumers [8]. Spam review threats have actually increased since anyone can just write and share spam reviews online with no restrictions. Some manufactures may hire persons for their items and services to compose fake reviews to fame their products. These persons are known as spammers. Fake reviews are typically published to gain and make profits, as well as to promote online services or products. This case is called a spamming review [9, 10]. According to existing studies, no effective method can discriminate between the features of truthful and deceptive reviews. Acquiring credible and comprehensive review website is the main objective of deceptive review detection methods, which filter the text content from deceptive and unwanted reviews. “Credibility” is a principle of great importance for opinion-mining applications. Credibility includes how stable and credible the intended system is. Thus, deceptive review identification methods are important for deleting and filtering deceptive reviews. The following is a condensed list of the contributions that may be drawn from this body of research:

1. Analyzing and detecting online deceptive reviews in electronic product reviews on Amazon and Yelp platforms.
2. Proposing an enhanced framework for online fake/deceptive feature reviews.
3. Proposing novel features, such as authenticity and analytical thinking that are used to differentiate between online fake and truthful reviews.
4. Labeling the Amazon review dataset based on extracted semantic and linguistics features from the review text.
5. Comparing and analyzing the results of the recurrent neural network (RNN, bidirectional long-short memory) model on the two datasets.

## 2. Challenges

There are a number of obstacles that must be overcome in order to spot fraudulent or fabricated reviews; some of the most prominent of them are as follows.

### 2.1. Less Awareness of the Features Associated with Deceptive/Fake/Spam from Several Different Types

The fake-correlated attributes are considered the main signs to effectively identify fake reviews of provided review text [11]. Some of the existing deceptive review detection studies utilize spam-related attributes particularly in application dimensions, including textual and behavioral dimensions [12, 13]. Additionally, almost all of the previous fake review identification researches have used a small number of attributes for fake review detection that reduces the performance in these systems [14]. Accordingly, a hybrid collection of features adopted must be defined from various genres, such as textual, behavioral, ranking, ordinal, and positional genres.

### 2.2. Difficulty in Applying Fake/Spam Review-Related Features to Preferences

Preference-based rating of spamicity attributes can be considered as one of the most important problems in deceptive/fake/spam review identification. Given that the significance of the value measurement of various features related to fake identification is difficult to determine, previous studies over a preference-based rating of fake features are relayed on graph representations [15–17]. Nevertheless, these methods are less effective when various collections of features are utilized [18]. Thus, effective techniques are required to classify features according to their preferences/significance in a specific e-domain.

### 2.3. Less Focus Is Paid to Creating a Cohesive Framework for the Identification of Reviews as Deceptive or Truthful

Previous studies on spam/fake detection, such as those reported by [19–21], concentrated on some basic aspects of review spamming and paid less emphasis on providing a coherent structure for the detection of fake reviews. Therefore, further work is needed to develop a coherent structure that can identify and categorize the review text as either deceptive or truthful.

## 3. Related Works

In this chapter, an analysis of previous works undertaken on the identification of deceptive/fake reviews is introduced. It also discusses the effective techniques and methods used in recent studies. Deceptive reviews have been identified as an apprehension for Internet marketing because they distress consumers' purchase decisions and therefore gain a comparative advantage. Supportive and harmful fake reviews are expected to fame or defame aimed products [22], as customers have a restricted capability and logic to analyze fake reviews [23, 24]. However, machine learning and deep learning techniques have been established to ascertain their rapid recognition on online shopping websites.

### 3.1. Linguistic Feature-Based Fake Review Identification

They proposed the first study regarding the issue of identifying opinions [25]. To identify opinion spam, they defined three kinds of reviews: untrue review, brand review, and nonreview. They used the logistic regression technique for the categorization of online customer's reviews into fake and truthful. Untrue reviews can be tough to detect because spammers typically turn their own reviews and evade detection by automatic methods. Through the Amazon review dataset, their methodology obtained 78% accuracy.

They leveraged Amazon Mechanical Turk (AMT) platform to create the experiment datasets and use a natural language understanding technology to mine linguistic features from review content [26]. They tested and compared a variety of classifiers. However, the findings achieved on actual AMT datasets were unsatisfactory.

They manually constructed fake review datasets from the Amazon website and then used the Naive Bayes machine learning technique to categorize the reviews into fake and truthful based on textual features [27]. In labeling a large number of unmarked reviews, a two-aspect cotraining semisupervised learning approach was introduced. Moreover, they utilized it as an evaluation dataset. The supervised methods presented by Radulescu [2] to detect fake reviews have three main processes: extraction of features, extraction of topics, and similarity of posted reviews. Based on YouTube reviews and daily graph news, they conducted the first two processes. The process was tested to understand the contextual relationship between the review text and the topic of the review, which determines whether the review text associates with the topic or not. Finally, they used three different classifiers to complete the classification task: Naive Bayes, decision tree, and support vector machine. According to the findings of the experiments, the decision tree method outperforms other classifiers, achieving 95 percent precision and 83 percent recall. Feng et al. [27] claimed that, in fraudulent review analysis, detailed syntactic aspects of the review text are extremely successful, and they used probabilistic context-free terminology (PCFT). The PCFT syntax-analyzing tree's conceptual principles are used to retrieve the deep lexical properties of the review contents. Fake reviews were detected using the SVM algorithm. Using the Amazon dataset, in [28] a deep feedforward neural network and a convolutional neural network were constructed for deep learning. A number of feature sets, including word emotions and N-grams, were employed. The deep feedforward neural network and convolutional neural network (CNN) techniques have accuracy ratings of 82 percent and 81 percent, respectively, according to the results. Ren et al. [21] proposed a hyper-deep learning model that consists of a gated RNN and CNN (GRNN-CNN) in detecting deceptive opinion spam. They used doctor, restaurant, and hotel datasets with sizes of 432, 720, and 1,280 reviews, respectively. By combining all of these datasets, they applied their proposed method for the classification of reviews into spam and nonspam reviews. The best classification result obtained was 83% accurate. Hussain et al. [29] used various supervised machine learning techniques for fake review detection using the Amazon dataset. They applied support vector machine, Random Forest, Naive Bayes, and logistic regression classifiers based on N-gram features. Based on the performance assessment, logistic regression performed better than other classifiers using unigrams, as well as bigram features, which achieved 88% accuracy.

### 3.2. Behavioral Feature-Based Fake Review Detection

Fake review identification using fraudulent behavioral characteristics is the discovery of uncommon behaviors and fraudulent relationships. At present, only a few researchers have analyzed the identification of spam detection by retaining spammer behavioral features. Mukherjee et al. [28] proposed a spam review detection approach utilizing a clustering method by analyzing spam reviews to classify the clusters into spammers and nonspammers. Heydari et al. [30] also presented a model that integrates only a certain reviewer's time series attributes on an actual Amazon dataset. They claimed that spammers cooperate in a group, and their main aim is always to promote or disrepute online products or services. Spammers are a group of people with the same IDs or with separate ID accounts. suggested a novel graph-based approach for detecting spammers in e-commerce websites using the Amazon dataset (1,950 reviews and reviewers). They investigated three different types of features: strong positive or negative, similarity rating, and average rating features. The experimental result of their methodology was 82% accurate.

Barbado et al. [31] offered outlines for review spammer recognition based on user-centric features. In their research, the authors focused on four different features: personal features, review activities, social features, and trust features. They evaluated the Yelp product review dataset with various supervised machine learning techniques, such as RF, LR, DT, Ada Boost, and NB. Based on the experimental results, Ada Boost has provided better performance than other algorithms, with an obtained accuracy of 82%.

## 4. Enhanced Framework for Textual and Behavioral Features for Deceptive/Spam/Fake Review Identification

Figure 1 presents an enhanced framework of textual and behavioral features for deceptive/fake/spam review identification. Strong positive and negative words are textual features that indicate whether a given review was written to fame or defame directed goods or services. A review rating is a value ranging from 1 to 5, as posted by the reviewer to rate a specific product or service. The reviews count represents the total amount of reviews that were posted by a reviewer. AS spammers have an intelligent way of writing spam reviews; therefore, based on the analytical thinking feature, we can calculate and analyze the degree of spammer's thinking. Authenticity is a textual feature used to differentiate between true teller reviewer (nonspammer) and liar reviewer (spammer). We assigned 50% as the threshold value for the authenticity feature. This value indicates that if the review text has attained ≥50%, it is labeled as truthful; otherwise, it is a deceptive review. An IP address is a behavioral feature used to identify the location of the reviewers where the reviews were posted. Additional details about these features are presented in Table 1 in Section 5.1.

## 5. Materials and Methods

Figure 2 presents the general framework planned for this methodology, which consists of seven modules: datasets, preprocessing, feature extraction, deep bidirectional long short-term memory technique, data splitting, performance assessment, and results. The components of the framework are described further below.

### 5.1. Datasets

Presented below are the datasets used in this research to identify deceptive/fake reviews. We compared the results from two datasets that were about the same in size.

#### 5.1.1. Yelp-Based Dataset

The Yelp-based dataset is a standard deceptive product review combined from four USA cities and used in a study presented by [32]. The Yelp filtering method used by Yelp.com [33] was used to label this dataset. There are 30,476 reviews and reviewers in the dataset, with attributes including rating value, reviewer name, confirmed purchase (Yes or No), reviewer ID, product ID, review title, and review text, as well as the class label. The dataset's range is depicted in Table 2.

#### 5.1.2. Amazon-Based Dataset

From 1996 to 2014, McAuley et al. (2015) compiled an Amazon-based dataset of 142.8 million product reviews. Rating value, reviewer ID, product ID, review title, and review text are all included in the dataset. Unlabeled cell phone and accessory characteristics were retrieved from the review text and utilized in a linguistic inquiry and word count (LIWC) program to provide a deceptiveness score (Equation 2) to a subset of this unlabeled dataset. The dataset used consisted of 30,471 reviews and reviewers. The distribution of the dataset is shown in Table 3.

For labeling, we extracted a set of significant features from the product's review text. These features are authenticity, analytical thinking, positive words, negative words, personal pronouns, negation words, comparing words (superlative and comparative adjectives), and sentiment scores, which are demonstrated in Table 1.

A deceptiveness score is the degree or measurement of deceptive hints and clues for a set of behavioral and linguistic features extracted from Amazon product review datasets wherein the review is labeled as either truthful or deceptive. In this approach, certain features are computed from the given product review that has been written by the reviewer. As shown in Table 4, each feature calculated its average and weight values.

To calculate deceptiveness score, we manually assigned each feature a weight value according to its average value. On the other hand the feature with the maximum average value will be assigned the highest weight value because of its contribution in the dataset. However, the deceptiveness score was obtained using the following equation:

(1) $$\begin{array}{c} DS\left(r\right)=\frac{\sum Fi\times Wi}{K}, \end{array}$$

where *DS*(*r*) signifies the deceptiveness score of the review *r*, *Fi* represents the feature value, *Wi* is the weight value given for the feature, and *K* is the total number of all features of the dataset.

After calculating the deceptiveness score using (1), we then normalized the deceptiveness score using the minimum maximum normalization approach and obtained a range of [0–1]. After normalization, a review text is labeled truthful or deceptive based on the threshold value represented by *T* = 0.50. Equation (2) is given for the review labeling process as follows:

(2) $$\begin{array}{c} {\text{Review}}_{\text{Label}}=\left\{\begin{array}{c} {\text{Review}}_{\text{truthful}},\text{if }SC\left(r\right)<T\\ {\text{Review}}_{\text{deceptive}},\text{if }SC\left(r\right)\geq T \end{array}\right.. \end{array}$$

### 5.2. Preprocessing

We performed the preprocessing steps on both datasets used. The data preprocessing phase has the goal of making the text presentable and easy to handle. The subsequent processes were carried out on the fully utilized datasets for this purpose.

#### 5.2.1. Lowercase

This is the method of transforming the review text's entire words to lowercase words.

#### 5.2.2. Stop Word Removal

Stop words are a group of commonly used terms in a language that have been eliminated from the evaluation since they do not contain any meaningful data for the model. Stop word occurrences are, for example, “the,” “a,” “an,” “is,” “are,” and so on.

#### 5.2.3. Punctuation Removal

Punctuation marks are to be removed from the review text as a part of this process.

#### 5.2.4. Removing One-Word Review

This task is used to remove one-word textual reviews.

#### 5.2.5. Removing Contractions

Replace a term written in the abbreviated form with its longer version. “When've” becomes “when have,” for example.

#### 5.2.6. Tokenization

Breaking sentences into smaller bits of words or tokens is the goal of this strategy.

#### 5.2.7. Padding Sequences

The input data for deep learning algorithms is always the same length, whether it is used for text categorization or other tasks. Afterwards, we applied the padding sequence strategy to limit the review to 250 words.

### 5.3. Extraction of Features Set and Analysis

Feature extraction is the third step in our proposed methodology and aims to extract a set of significant features from the review text. For this purpose, we input all review texts of both datasets into the LIWC tool and extracted specific linguistic features from the plain text. LIWC is defined as a computer program-based text analysis that produces more than 90 variables as outputs. It is used to analyze and compute important features from a given text individually. We utilized some of the LIWC's output variables as a feature set to distinguish between deceptive and truthful reviews in the Amazon dataset and for the analysis of the Yelp dataset.

### 5.4. Data Splitting

This module presents the division of the different datasets used in the experiments. After we labeled an Amazon dataset based on the previously described extracted features, we divided each utilized dataset for the training, testing, and validation of the proposed deep bidirectional long short-term memory (DBiLSTM) model, as depicted in Table 5.

### 5.5. Deep Bidirectional Long-Short Memory-Based Deceptive/Fake Reviews Identification

RNN is a form of deep learning neural network employed in various domains, such as medical image diagnosis, pattern recognition, natural language processing, and computer vision and so on. Compared with different deep artificial neural networks, the RNN has a steering control loop, which assists in the preservation, recollection, and addition of early states to the existing output. One issue in the RNN network is the gradient disappearing point [34–37]. To sort this issue, the LSTM model has been presented [38–45]. Memory units in LSTM can ultimately carry the results from past data samples *X* into the prediction of *Y*. Furthermore, the processing of data training occurs in one direction—only on a forward direction which neglects the backward connection and causes the system to be less efficient. To overcome this drawback, the data training phase in a bidirectional long-short memory system is performed in forward and backward directions. There are four gates in the LSTM unit: input *i*_*t*_, forget *f*_*t*_, cell state *c*_*t*_, and output gate *o*_*t*_. This feature improves the performance of the system.  Figure 3 illustrates the structure of bidirectional LSTM for review text representation.

Let the review text *R* consist of a group of words *W*_*n*_, indicating that *R* = (*W*_1_, *W*_2_,…, *W*_*n*_); then each word will be embedded to its real value vector using a word embedding layer that is one layer of the used model. Additional details about this layer are shown in Section B. Each LSTM unit has four gates, as depicted in equations (2)–(5).

(3) $$\begin{array}{c} i_{t}=\sigma \left(W_{ix}x_{t}+W_{ih}h_{t-1}+b_{i}\right), \end{array}$$

(4) $$\begin{array}{c} f_{t}=\sigma \left(W_{fx}x_{t}+W_{fh}h_{t-1}+b_{f}\right) \end{array}$$

(5) $$\begin{array}{c} o_{t}=\sigma \left(W_{ox}\right.x_{t}+W_{oh}h_{t-1}+b_{o}\; \end{array}$$

(6) $$\begin{array}{c} c_{t}=f_{t}c_{t-1}+i_{t}*\;\tanh\left(\;W_{cx}x_{t}+W_{ch}h_{t-1}+b_{c}\right)\; \end{array}$$

where *x* is the input sequence vector; *i*_*t*_, *o*_*t*_ refer to input, output gates; and *f*_*t*_ is the forget gate that is used to filter the unrequired information. tanh and *σ* are the activation functions, and *b* and *W* represent biased and weight factors, respectively. *c*_*t*_ and *c*_*t*−1_ are the updated and outdated states of a memory cell, respectively. The forget gate *f*_*t*_ drives how much outdated information must be disregarded, whereas the input gate *i*_*t*_ controls the amount of information that must be kept. The memory cell  *c*_*t*_ is distributed over a tanh activation function and organized through the output gate *o*_*t*_, which directs information presented in the memory cell to be passed to the output, as expressed in (5).

(7) $$\begin{array}{c} \overset{⟶}{\;h_{t}}=o_{t}*tanh\left(c_{t}\right),\\ tanh\left(x\right)=\;\frac{\;1-e^{2x}}{\;1-e^{2x}}, \end{array}$$

(8) $$\begin{array}{c} H_{t}=\left(\overset{⟶}{\;h_{t}}\;∶\overset{\leftarrow }{\;h_{t}}\right). \end{array}$$

where *H*_*t*_ represents yielding of the bidirectional concatenation of $\overset{⟶}{\;h_{t}}$ forward and $\overset{\leftarrow }{\;h_{t}}$ backward LSTM units at the existent time *t*. The memory cell and gate structure mechanism efficiently provide a solution to the issue of a disappearing gradient and an explosion slope of RNN. Therefore, LSTM can abstract the long-distance holding of sequences mining. Corresponding to a normal LSTM, the bidirectional LSTM [46–49] can extract bidirectional sequence data from the input sequence.  Figure 3 shows the process of RNN bidirectional long-short memory model. Furthermore, it transfers input sequences from two directions to one output direction in the networks as presented in Figure 4.

Figure 4 displays a comprehensive construction of the planned model in detecting and classifying the fake/deceptive reviews by using two different domain datasets from the Amazon and Yelp platforms. The definitions and descriptions of every component and layer used in the above model are as follows:

(A) Input layer: This is the first layer of the proposed BiLSTM model utilized that accepts the preprocessed data and specifies the input length in this model that represents the count of words for the maximum review text length, which is equal to 250 words.
(B) Embedding layer: This layer works only in natural language text processing and is the initial hidden layer in the neural network (Cho et al. [35]). In our proposed model, an embedding layer was used to randomly provide weights for words in the training data. This means each word embedding is furthered as an input (review text matrix) to the bidirectional LSTM layer. An embedding layer in this model consists of three modules with assigned values: the maximum features are assigned to 50,000 words; the word embedding dimension size of the vector is allocated to 100 dimensions, which by each word in the sentence of the review text will be embedded; and the input sequences length is given to 250 words. The subsequent yield of an embedding layer is represented in a two-dimensional vector space that concludes the embedding for all the words existing in the training data.
(C) Bidirectional LSTM: This consists of two opposite direction layers employed to receive the vector of input sequences from the previous layer and begins with the handling process. We used 100 hidden units of LSTM for the training sequence process. Forward and backward LSTM layers represent bidirectional LSTM. The working theory is that the forward layer catches the sequence's historical data, which is the past data, whereas the backward layer catches the sequence's future information. These two layers are concatenated to form one output. The main highlight of this architecture is that knowledge about the sequence meaning is thoroughly considered.
(D) Dense layer (fully connected layer): This layer is comprised of *N* artificial neurons. The main task of this layer is to connect all neurons together in the network and handling the sequences information and forwarding them to the succeeding output layer. The activation function implemented by this layer is a rectified linear unit which is expressed in the following equation:
  (9) $$\begin{array}{c} f\left(x\right)=\max\left(0,x\right). \end{array}$$
(E) SoftMax activation function: This is the last layer applied in the BiLSTM model used for the classification of output classes of the evaluated datasets. The number of neurons in this layer is set based on the number of classes in the dataset. Furthermore, it is its activation function that performs calculations of probability distribution for the input sequences vector of the reviews texts of the used dataset. An equation for the SoftMax activation function is expressed mathematically as follows:
  (10) $$\begin{array}{c} \sigma \left(z\right)=\frac{e^{z_{i}}}{\sum_{j=1}^{K}e^{z_{j}}}, \end{array}$$
where *z* denotes the values of the neurons placed in the output layer. An *e* is exponential that acts as nonlinear function.

Table 6 summarizes the hyperparameters used in the bidirectional LSTM model.

Each epoch indicates the number of iterations of forward and backward passes for training samples that can be considered to the DBiLSTM model. The batch size acts as the number of training samples that were taken each iteration. The dropout is hidden layer and was applied to prevent an overfitting problem in the model' performance.

### 5.6. Performance Evaluation Metrics

In terms of False Positive and False Negative rates, we can assess how well the proposed model can categorize and discriminate among deceptive and truthful review texts. We used a variety of performance evaluation metrics to evaluate the BiLSTM model's classification accuracy. The following are the definitions and equations of these metrics:

(11) $$\begin{array}{c} \;Accuracy=\frac{TP+TN}{FP+FN+TP+TN}\;\times 100, \end{array}$$

(12) $$\begin{array}{c} Precision=\frac{TP}{TP+FP}\;\times 100, \end{array}$$

(13) $$\begin{array}{c} \;Sensitivity=\frac{TP}{TP+FN}\;\times 100, \end{array}$$

(14) $$\begin{array}{c} \;specificity=\frac{TN}{TN+FP}\;\times 100, \end{array}$$

(15) $$\begin{array}{c} \;F1-score=2*\frac{precision\;\times \;sensitivity}{precision+\;sensitivity}\;\times 100. \end{array}$$

The TN stands for true negative, and it shows the total number of samples correctly classified as misleading reviews. The total number of samples incorrectly classified as truthful reviews is known as False Negative (FN). The total number of samples accurately categorized as truthful reviews is known as True Positive (TP). The total number of samples wrongly classified as deceptive reviews is known as False Positive (FP). In confusion matrices showed in Figures 5 and 6, zero (0) and one (1) indicate the deceptive and truthful review classes, respectively.

## 6. Experimental Results and Discussion

On the basis of the learning of word embedding of the review text, deep BiLSTM model was applied for deceptive review identification. In this study, two experimentations works were performed on two diverse datasets. The first one was executed on the standard Yelp product reviews and the second one on unlabeled Amazon product reviews. For the Amazon dataset, we labeled it using deceptiveness score calculations based on linguistic and behavioral features mined from the review text by the LIWC program. These features were authenticity, analytical thinking, positive words, negative words, comparing words, and negation words. We implemented the proposed model on the Yelp and Amazon datasets. The results obtained from these experiments were executed to examine the effectiveness of the model on the datasets used. The important role of the used model is to categorize the review text as a deceptive or truthful review. By comparing the testing results, we observed that BiLSTM provided similar testing accuracy in both datasets. With respect to the Yelp dataset, the model provided satisfactory results for sensitivity and F-score measures, whereas in the case of the Amazon dataset, the model showed improved results for precision and specificity measures.  Figure 7 shows the visualization of the classification results for both datasets.

After investigating the results obtained by authenticity (this feature calculates the truthfulness of the written review text) and analytical thinking (this feature analyzes the thinking of a reviewer) features, we found that these features proved their efficiency in differentiating between deceptive and truthful reviews.  Figure 8 shows the visualization of the average values of authenticity and analytical thinking in the Amazon and Yelp datasets.

The training and validation performance of the DBiLSTM model are presented in Figure 9. This shows that the training process reached 92%, whereas the validation process reached 89% with 50 epochs in the Yelp dataset. The performance of the proposed system showed good accuracy on the Amazon dataset. The training and validation accuracy rates reached 94% and 90%, respectively.

The accuracy loss of the proposed system is presented in Figure 10. The training and validation loss of the DBiLSTM model on the Yelp dataset decreased to 0.2 with 50 epochs, and the accuracy loss of the proposed system on the Amazon dataset also decreased.

### 6.1. Word Cloud

A word cloud is defined as the visualization tool for the most frequently repeated words in a given review text. Figures 11 and 12 show the word cloud for fake and truthful reviews in the Amazon dataset.

## 7. Comparative Analysis with Existing Approaches

Table 7 summarizes and presents a comparison of the accuracy attained by the proposed model with existing research work.

By comparing the results of our suggested model with some existing methods, such as the method presented by Barbado et al. [31], we concluded that the BiLSTM neural network with LIWC features and word embedding improved the accuracy rate for deceptive review detection. This result is because each word in the review text was transformed into multi-n-dimensional (100 dimensions) vector representations, and this feature makes the model learn the relationship between words in the training data. By contrast, the term frequency-inverse document frequency can only transform each word into a single-dimensional representation vector.

## 8. Conclusion

Given the current potential influence of deceptive reviews on customer's behavior and decision making in acquiring products or services, deceptive review identification has attained important considerations in both academic research and e-business fields. In this study, we attempted to solve the problem of deceptive reviews present in electronic product reviews on the Amazon and Yelp platforms based on linguistic and behavioral features. As presented in this study, the detection of deceptive reviews contents by reading them remains a difficult task for humans. Therefore, investigating a set of review and reviewer features in identifying deceptive and truthful reviews is important for e-commerce plans and customers' purchasing decisions to select their favorite product. The exploration of the result values obtained by authenticity and analytical thinking features proved their proficiency in distinguishing between deceptive and truthful reviews in the Amazon and Yelp datasets. Through statistical evaluation, we discovered a difference between the average values of authenticity and analytical thinking scores in the Amazon and Yelp datasets. In the case of the Amazon dataset, the average authenticity scores for the deceptive and truthful reviews were 14.16% and 80.59%, respectively. In the Yelp dataset, the average authenticity scores for the deceptive and truthful reviews were 30.57% and 75.40%, respectively. Regarding the average value for the analytical thinking feature, in the Amazon dataset, the deceptive and truthful reviews exhibited 58.47% and 51.55%, respectively, and in the Yelp dataset, the deceptive and truthful reviews were 66.62% and 42.59%, respectively. By comparing the classification results of these experiments, we observed that the DBiLSTM model provided similar testing accuracies in both datasets. In the Yelp dataset, the model provided improved results for sensitivity and F-score measures, and in the Amazon dataset, the model provided satisfactory results for precision and specificity measures. The results presented in this research work suggested that the proposed DBiLSTM model can be used in associated text classification, such as fake news detection. Another conclusion of this research work and related works on deceptive review detection is that no large-scale labeled dataset exists for training the machine learning classifier. In future works, we will attempt to consider combining all review, reviewer, and product-centric features in developing a model for deceptive review identification in the online e-commerce platform [50, 51].

## Figures and Tables

**Figure 1:** Enhanced framework for deceptive/fake/spam review identification.

**Figure 2:** The framework of suggested method.

**Figure 3:** Working of the bidirectional long short-term memory model for learning review text representation.

**Figure 4:** Complete construction of the used model.

**Figure 5:** Confusion matrix for the Yelp dataset.

**Figure 6:** Confusion matrix for the Amazon dataset.

**Figure 7:** Visualization of testing results of the proposed model.

**Figure 8:** Visualization of an average value for analytical thinking and authenticity features in the Amazon and Yelp datasets.

**Figure 9:** Training and validation accuracy for the Yelp dataset (a) and Amazon dataset (b).

**Figure 10:** Training and validation loss of the deep bidirectional long short-term memory model for the Yelp (a) and Amazon (b) datasets.

**Figure 11:** Word cloud for deceptive reviews.

**Figure 12:** Word cloud for truthful reviews.

**Table 1:** Summary of selected textual and behavioral features with their equations for deceptiveness score calculation for labeling the product reviews of the Amazon dataset.

Feature ID	Explanation	Formula	Review example	Interpretation
*F*1	Proportion of strong positive words in the review content.	*F*1=*NPW*/*RL∗*100 NPW denotes a number of positive words. RL refers to the length of the review content.	“I love this charger; it has two ports for my phone and iPod. Sleek and convenient to store, and I just love it.	It indicates the review contents are strongly positive and plays an important function in spamicity calculation (Jindal et al. [6]).
*F*2	Proportion of strong negative words in the review.	*F*2=*NNW*/*RL∗*100 NNW states the number of negative words. RL refers to the length of the review content.	“I am disappointed that the 1A did not work with my iPad. That is what I get for buying a cheap adapter.”	This feature specifies whether the review contents are strongly negative or not and can help in the calculation of spamicity (Jindal et al. [6]).
*F*3	Percentage of numbers utilized in the review contents.	*F*3=*N*/*RL∗*100 *N* refers to number of numeric digits utilized in the review content.	“I have **8** chargers. I have more than **4** vehicles, so I keep more than **1** of these in each.”	Increased utilization of numbers indicates that the review text is so specialized; thus, the review is regarded as a nonreview (Jindal et al. [6]). This review is a type 3 fake review.
*F*4	Reviewer's writing authenticity.	Authenticity = ∑ PP + IP + excl (differ)−Negemo–Motion (5) This formula represents the total percentage of personal and impersonal pronouns, negative emotion words, and exclusive words in the review contents. We considered 50% to be a threshold value for this feature. Truthful review is ≥50%, whereas fake review is <50%.	“Surprisingly, this inexpensive version works just as well and just as reliably as the expensive variety. It has been working for me for months now. No problem. Excellent value.”	This feature shows the authenticity of reviewer writing. It is used to differentiate between true teller reviewers (nonspammer) and liar reviewers (spammer) (Newman et al. 2003). It has a score ranging from 1 to 100. The review mentioned in a neighbor cell has a 3.8% authenticity score; thus, it is tagged as a deceptive review.
F5	Analytic thinking of the reviewer.	Analytic thinking = ∑30 + articles + prep − PP − IMP − auxverb − conj − adverb − Negation. Articles, prep, PP, IMP, auxverb, conj, adverb, and negation represent the total percentage of articles, prepositions, personal pronouns, and impersonal pronouns in addition to auxiliary verbs, conjunctions, adverbs, and negation words in the text review.	“It worked great for the first couple of weeks, then it just stopped completely. So basically a small waste of money.” The above review has 68.29% analytic thinking value. It is tagged as a fake review.	This feature was used to calculate the analytic thinking of the reviewer. Spammers have an intelligent way of writing spam reviews. Based on the mentioned feature, we calculated and analyzed the degree of spammer's thinking. It has a value ranging from 1% to 99% (Pennebaker et al. 2015).
*F*6	Percentage of comparative words that the reviewer used in the review text.	*F*6=*CW*/*RL* CW denotes the percentage of comparing words, and RL is the review length. Comparing words is like comparative and superlative adjectives in the review content.	“Samsung mobile chargers are of higher quality and durability than Huawei mobile chargers.”	This feature acts as the count of the superlative and comparative adjective words. It shows the comparison between the two entities. Such text written by the reviewer is labeled as a spammer.

**Table 2:** Distribution of the Yelp dataset.

City name	Fake reviews	Truthful reviews
Los Angeles	6,270	6,009
Miami	1,696	1,767
New York	3,865	3,979
San Francisco	3,642	3,248

**Table 3:** Distribution of the Amazon dataset.

Description	Number of reviews and reviewers
Mobile decorative stickers	8,050
Mobiles back casing	6,171
Mobiles chargers	7,100
Mobiles batteries	9,150

**Table 4:** List of features extracted from the Amazon dataset with their average and weight.

Feature ID	Feature name	Average value	Weight
F1	Analytical thinking	82.07	0.9
F2	Authenticity	31.50	0.8
F3	Review length	22.41	0.7
F4	Rating value	3.63	0.3
F5	Comparing words	3.09	0.2
F6	Numeric digits	1.01	0.1
F7	Positive sentiment words	0.341	0.1
F8	Negative sentiment words	0.083	0.1

**Table 5:** Dividing of the evaluated datasets.

Dataset name	Count of samples	Training set (60%)	Testing set (20%)	Validation set (20%)	Count of deceptive class	Count of truthful class
Yelp	30,476	19,504	6,096	4,876	15,473	15,003
Amazon	30,471	19,500	6,095	4,876	15,753	14,718

**Table 6:** Parameters and their values used in the bidirectional LSTM model.

Parameter name	Value
Bidirectional LSTM units	100
Drop out layer	0.2
Dense layer	256
SoftMax layer	2
Epochs	5
Batch size	60

**Table 7:** Comparison results based on accuracy metric.

Paper	Dataset used	Features used	Technique	Accuracy (%)
Barbado et al. [31]	Yelp's product review dataset	Term frequency-inverse document frequency and sentiment score features	Adaptive boost BiLSTM	82
Proposed work	Yelp' product reviews dataset	LIWC features and word embedding (Word2Vec)	BiLSTM	**89.6**

## Data Availability

Authors have picked up the dataset from https://www.sciencedirect.com/science/article/abs/pii/S030645731730657X.
